The article "Using Fuzzy Logic Techniques for Assertion-Based Software Testing Metrics" was published in 2015. Journal: ScientificWorldJournal.

# Using Fuzzy Logic Techniques for Assertion-Based Software Testing Metrics

**DOI:** 10.1155/2015/629430

**Published:** 2015-04-28

**Authors:** Ali M. Alakeel

**Affiliations:** College of Computers and Information Technology, University of Tabuk, P.O. Box 1458, Tabuk 71431, Saudi Arabia

## Abstract

Software testing is a very labor intensive and costly task. Therefore, many software testing techniques to automate the process of software testing have been reported in the literature. Assertion-Based automated software testing has been shown to be effective in detecting program faults as compared to traditional black-box and white-box software testing methods. However, the applicability of this approach in the presence of large numbers of assertions may be very costly. Therefore, software developers need assistance while making decision to apply Assertion-Based testing in order for them to get the benefits of this approach at an acceptable level of costs. In this paper, we present an Assertion-Based testing metrics technique that is based on fuzzy logic. The main goal of the proposed technique is to enhance the performance of Assertion-Based software testing in the presence of large numbers of assertions. To evaluate the proposed technique, an experimental study was performed in which the proposed technique is applied on programs with assertions. The result of this experiment shows that the effectiveness and performance of Assertion-Based software testing have improved when applying the proposed testing metrics technique.

## 1. Introduction

Software testing is a very labor intensive and costly task. Theretofore, many software testing techniques to automate the process of software testing have been reported in the literature, for example, [1–8]. There are two main approaches to software testing: black-box and white-box [9]. Test data generation is the process of finding program input data that satisfies a given criteria. Test generators that support black-box testing create test cases by using a set of rules and procedures; the most popular methods include equivalence class partitioning, boundary value analysis, and cause-effect graphing [9]. White-box testing is supported by coverage analyzers that assess the coverage of test cases with respect to executed statements, branches, paths, and so forth. Programmers usually start by testing software using black-box methods against a given specification. By their nature black-box testing methods might not lead to the execution of all parts of the code. Therefore, this method may not uncover all faults in the program. To increase the possibility of uncovering program faults, white-box testing is then used to ensure that an acceptable coverage has been reached, for example, branch coverage.

The article "Using Fuzzy Logic Techniques for Assertion-Based Software Testing Metrics" was published in 2015. Journal: ScientificWorldJournal.

It has been reported in [4] that Assertion-Based software testing is effective in detecting program faults as compared to traditional black-box and white-box software testing methods. The main goal of Assertion-Based testing [4] is to find a program input on which an assertion is violated. If such an input is found then there is a fault in the program. Some programming languages support assertions by default, for example, Java and Perl. For languages without built-in support, assertions can be added in the form of annotated statements. In [4], assertions are represented as commented statements that are preprocessed and converted into Pascal code before compilation. Many types of assertions can be easily generated automatically such as boundary checks, division by zero, null pointers, and variable overflow/underflow. Therefore, programmers may be encouraged to write more assertions in their programs in order to enhance their confidence in their programs.

Although Assertion-Based testing is a promising approach in terms of detecting program's faults, the applicability of this approach in the presence of larger numbers of assertions may be costly. This cost is related to search time required for finding a test data to violate such a large number of assertions which may hamper the effectiveness of Assertion-Based testing and makes it impractical for industrial-size software. Therefore, software developers testing need to decide when to apply Assertion-Based testing in order to get the benefits of this approach at an acceptable level of costs. In this paper, we present an Assertion-Based testing metrics technique that is based on fuzzy logic techniques [10]. The main goal of the proposed technique is to enhance the performance of Assertion-Based software testing in the presence of large numbers of assertions. Additionally, this technique may assist software developers to get the most benefits of Assertion-Based testing. More specifically, our objective is to assist software developers while making their decision to apply Assertion-Based testing method to their software. Furthermore, given a program to be tested, this research provides the developer with an estimation of the required level of details necessary to test this program using Assertion-Based software testing. By level of details we mean the number of assertions that will be explored for violations. The results of applying the proposed technique for Assertion-Based testing metrics may save valuable testing resources during the process of software testing.

The rest of this paper is organized as follows. Assertion-Based testing is presented in Section 2. In Section 3, related work is discussed. We present our approach for Assertion-Based testing metrics in Section 4. An experimental study is presented in Section 5 and our conclusions and future work are discussed in Section 6.

The article "Using Fuzzy Logic Techniques for Assertion-Based Software Testing Metrics" was published in 2015. Journal: ScientificWorldJournal.

## 2. Assertion-Based Software Testing

Assertions have been recognized as a powerful tool for automatic run-time detection of software errors during testing, debugging, and maintenance, for example, [11–17]. An assertion specifies a constraint that applies to some state of a computation. When an assertion evaluates to a false during program execution, this indicates an incorrect state in the program. Assertion-Based automated software testing [4] is an approach that employs program assertions for the purpose of test data generation. As reported in [4], Assertion-Based testing was able to uncover program faults which were uncovered by black-box and white-box testing.

Given an assertion *A*, the goal of Assertion-Based testing is to identify program input for which *A* will be violated. Assertion-Based testing is a goal-oriented approach [1–3] that is based on the actual program's execution. Assertion-Based testing reduces the problem of test data generation to the problem of finding input data to execute a target program's statement s. In this method, each assertion is eventually represented by a set of program's statements (nodes). The execution of any of these nodes causes the violation of this assertion. In order to generate input data to execute a target statement s (node), this method uses the chaining approach [3]. Given a target program statement s, the chaining approach starts by executing the program for an arbitrary input. When the target statement s is not executed on this input, a fitness function [2] is associated with this statement and function minimization search algorithms are used to find automatically input to execute s. If the search process cannot find program input to execute s, this method identifies program's statements that have to be executed prior to reaching the target statement s. In this way this approach builds a chain of goals that have to be satisfied before the execution to the target statement s. More details of the chaining approach can be found in [3].

The main aim of Assertion-Based software testing is to increase the developer confidence in the software under test. Therefore, Assertion-Based software is intended to be used as an extra and complimentary step after all traditional testing methods have been performed to the software. Assertion-Based testing gives the tester the chance to think deeply about the software under test and to locate positions in the software that are very important with regard to the functionality of the software. After locating those important locations, assertions are added to guard against possible errors with regard to the functionality performed in these locations.

The article "Using Fuzzy Logic Techniques for Assertion-Based Software Testing Metrics" was published in 2015. Journal: ScientificWorldJournal.

An assertion may be described as a Boolean formula built from the logical expressions and from the (**and**,** or**,** not**) operators. There are two types of logical expressions: Boolean expression and relational expression. A Boolean expression involves Boolean variables and has the following form: e1* op* e2, where e1 and e2 are Boolean variables or true/false constant and* op* is one of { = , ≠}. Relational expressions, on the other hand, have the following form: e1* op* e2, where e1 and e2 are arithmetic expressions and* op* is one of {<, ≤, >, ≥, = , ≠}. For example, (*x* < *y*) is a relational expression, and (*f* = false) is a Boolean expression.

As reported in [4], an assertion may be described as a Boolean formula built from the logical expressions and from (**and**,** or**,** not**) operators. In [7], Pascal language notation is used to describe logical expressions. There are two types of logical expressions: Boolean expression and relational expression. A Boolean expression involves Boolean variables and has the following form: A_1_ *op* A_2_, where A_1_ and A_2_ are Boolean variables or true/false constant, and* op* is one of { = , ≠}. On the other hand, relational expression has the following form: A_1_ *op* A_2_, where A_1_ and A_2_ are arithmetic expressions and* op* is one of {<, ≤, >, ≥, = , ≠}. For example, (*x* < *y*) is a relational expression, and (*f* = false) is a Boolean expression. For example, the following is a sample assertion:

 A: (^∗^@ (*x* < *y*)** and** (*f* = false) @^∗^),

which will be translated during a preprocessing stage [4] into the following code:

 if** not** ((*x* < *y*)** and** (*f* = false)),
 then Report_Violation;

where Report_Violation is a special procedure which is called to report an assertion's violation.  Algorithm 1 shows a sample Java method with assertions. This simple method computes the maximum and minimum element of a set of integers.

## 3. Related Work

One of the major problems faced during software testing is deciding when to stop the testing process [9]. This is very important because software developer would like to stop testing only after she has a certain level of confidence that more testing will not reveal faults in their software. Software testing metrics is the measurements of the effectiveness of a testing method on revealing program faults [18]. Most of existing software testing metric methods measure what effect an execution of a program's statement has on detecting program's faults, for example, [19–25]. With respect to Assertion-Based software testing, existing testing metric methods may be used to measure how much effect violating a single assertion has on uncovering program's errors. This is possible because each assertion is eventually transformed into one or more program's statements [4]. However, for programs with large numbers of assertions, estimating the effectiveness of applying Assertion-Based testing [4] when applied to test these types of software is yet to be measured. The contribution of the testing metrics approach presented in this paper is to formulate a method by which software developers are assisted while making their decision on the applicability of Assertion-Based testing to their software. This assistance is offered through utilizing the powers of fuzzy logic techniques [10] in directing Assertion-Based testing efforts toward those parts of the program that may need thorough testing. By doing so, the effectiveness of Assertion-Based testing is enhanced and valuable testing resources are invested wisely, which may lead to the detections of more programs' faults.

The article "Using Fuzzy Logic Techniques for Assertion-Based Software Testing Metrics" was published in 2015. Journal: ScientificWorldJournal.

## 4. Assertion-Based Software Testing Metrics

As stated in [4], Assertion-Based software testing is recommended to be applied to the software after traditional testing methods such as black-box and white-box have been applied. Therefore, the application of Assertion-Based software testing is an additional step to enhance software developers' confidence on their software correctness. Because the number of assertions may be very large for complex commercial software, the process of exploring all assertions may require a huge amount of search time. Additionally, development scheduling and delivery dates may not allow for the whole Assertion-Based testing process to be performed. The main goal of this research is to measure the applicability of Assertion-Based software testing to a given program. In other words, our objective is to assist software developers while making their decisions to apply Assertion-Based software testing method on their software. If Assertion-Based testing method is utilized intelligently, the chances of violating more assertions increase, therefore, detecting more programs' errors where this is the ultimate goal of software testing.

The proposed testing metrics approach works as follows. Give a program P with assertions, before applying Assertion-Based testing on P, and this approach starts by classifying the P units, that is, modules or procedures, based on two main criterions: importance and confidence. The main objective of the proposed approach is to make Assertion-Based software testing more efficient and effective. To satisfy this objective, more testing resources will be directed toward those parts of the program that need to be tested more. For example, a program unit that performs dynamic computations should more important than a graphical interface unit that displays the company's logo. Because it is difficult to quantify the notion of “importance” and “confidence,” we propose to utilize the powers of fuzzy logic techniques [10, 26]. The reason of choosing fuzzy logic to deal with these properties is the difficulty to draw crisp boundaries between program's units in our classification.

The article "Using Fuzzy Logic Techniques for Assertion-Based Software Testing Metrics" was published in 2015. Journal: ScientificWorldJournal.

At first, the proposed approach orders each program's unit according to their importance with respect to the functionality of the program under test. Using fuzzy logic terms, this classification is mapped into a single fuzzy set [10], named IMPORTANCE. The objective of this classification is to grade the importance of each program's unit with respect to the whole software under consideration. This will help developers making their decision on whether to invest more testing resources in a given program's unit or not.

In the next step, the proposed approach measures the confidence level of the developer in the correctness of each of the program's units. Given a program unit *U*, this step is achieved by asking each developer to specify a percentage value to express her confidence in the correctness of *U* based on her believes in the effectiveness of tests that were performed to test *U* previously. As with the issue of importance, it is very difficult to express a developer confidence level, in a certain unit *U*, within crisp boundaries agreeable by different people on various types of programs. Therefore, we create a fuzzy set named, CONFIDENCE, in order to capture a developer's confidence in the correctness of a given program's unit *U*.

For presentation purposes, let P be a program under consideration with units *U* = {*u*_1_, *u*_2_,…, *u*_*n*_}, where each unit, *u*_*k*_, has a number of program assertions: *A*_*uk*_ = {*a*_1_, *a*_2_,…, *a*_*m*_}. The application of the proposed approach for Assertion-Based software testing metrics on P proceeds as follows. First, all units of P are identified and classified according to their importance to the correctness of the program P. The result of this step is that each program's unit, *u*_*k*_, will belong to the IMPORTANCE fuzzy set with a certain membership degree. As mentioned earlier, because the notion of importance is subjective and may differ from one software to another and from a developer to another, we utilize the flexibility of fuzzy logic [10] in order to quantify the term “importance” of a program's unit. Therefore, in order to create the membership degree of a unit, we first asked the developers of the programs to rate the importance of their program's unit based on their own believe and experience. After that we used *S*-function [26], shown in (1), to map the data obtained from developers into a membership degrees to the fuzzy set IMPORTANCE. According to fuzzy sets rules [10], this membership degree is on the interval [0,1] and it reflects the compatibility of each program unit, *u*_*k*_, to the fuzzy set.

The article "Using Fuzzy Logic Techniques for Assertion-Based Software Testing Metrics" was published in 2015. Journal: ScientificWorldJournal.

The* S*-function is as follows:

(1) $$\begin{array}{c} S\left(x;\alpha ,\beta ,\gamma \right)=\left\{\begin{array}{cc} 0 & \text{for}\;x\leq \alpha \\ 2{\left(\frac{x-\alpha }{\gamma -\alpha }\right)}^{2} & \text{for}\;\alpha \leq x\leq \beta \\ 1-2{\left(\frac{x-\gamma }{\gamma -\alpha }\right)}^{2} & \text{for}\;\beta \leq x\leq \gamma \\ 1 & \text{for}\;x\geq \gamma . \end{array}\right. \end{array}$$

Given a set of programs units that were classified according to their importance, the second step of the proposed approach is to decide whether or not to apply Assertion-Based testing to these classified units. In order to make this decision, we need to estimate the developer's confidence on the correctness of each unit based on her experience with previous tests, for example, black-box and white-box, that were applied, previously, to test program P. As with the notion of “importance,” the notion of “confidence” is subjective and may differ from one person to another. Therefore, for the purpose of capturing developers confidence in the correctness of their programs, we asked them to express their confidence on the correctness of each program unit, *u*_*k*_, based on previous tests results applied to test *u*_*k*_. The data obtained from developers is mapped using the *S*-function to create each unit, *u*_*k*_, membership degree to the fuzzy set, CONFIDENCE, mentioned above with a certain membership degree, *u*_*km*_.

The *S*-function may be described as follows:

- a mathematical function that is used in fuzzy sets as a membership function;
- a simple but valuable tool in defining fuzzy functions such as the term “confidence”;
- rather than mainlining a table defining the membership function, all data may by compactly represented by a formula;
- *α*, *β*, and *γ* are parameters which may be adjusted to fit the desired membership data;
- the *S*-function is flat at a value of zero for *x* ≤ *α* and at 1 for *x* ≥ *γ*. In between *α* and *γ*, the *S*-function is a quadratic function of *x*. The *β* parameter corresponds to the crossover point of 0.5 and is (*α* + *γ*)/2.

In order to illustrate the functionality of the proposed technique, consider the following example. Let P to be the first program used in our experiment, “Boyer-Moore,” as shown in Table 1. This program has a total of four units: Unit_1, Unit_2, Unit_3, and Unit_4. In order to know the importance of these units with respect to the whole program, P, from the point of view of those developers who wrote the code of P, we polled the three developers who participated in writing three versions of P. We obtained the following data shown in Table 1.

The article "Using Fuzzy Logic Techniques for Assertion-Based Software Testing Metrics" was published in 2015. Journal: ScientificWorldJournal.

Using the “importance” data shown in Table 1, we construct the fuzzy set IMPORTANCE, using the *S*-function, as follows. In order to use the *S*-function, we have to find what values to be used for the parameters: *α*, *β*, and *γ*. Based on the data obtained from the developers regarding the importance of the units of this example program, we set the values of these parameters as

(2) $$\begin{array}{c} \alpha =10,\\ \gamma =100,\\ \beta =\frac{\left(\alpha +\gamma \right)}{2}=55. \end{array}$$

Note that, based on the properties of the *S*-function [26], the value of *α* represents the least value a program's unit may receive and the value of *γ* represents the most value a unit may receive. Specifically, the value of 10 for *α* parameter means that no unit of this specific program, P, is less than 10% of importance to the functionality of the whole program. Similarly, the value of 100 for *γ* parameter says that a unit may be extremely important to the functionality of P. Note that the values of *α* and *γ* parameters may be adjusted to fit the desired membership data. By plugging these values in the *S*-function of (1), the membership degrees for the four units of this example program to the fuzzy set IMPORTANCE are as follows:

 IMPORTANCE = {0.1/Unit_1, 0.54/Unit_2, 0.9/Unit_4, 0.98/Unit_3}.

From these values in the fuzzy function IMPORTANCE, the proposed approach deduces that Unit_3 and Unit_4 are the most important units of the program P. Therefore, more testing resources will be directed toward testing these units. In addition, these values indicate that Unit_2 is more important than Unit_1; therefore, more testing will be applied to violate assertions in Unit_2 as compared when testing Unit_1.

From this example, note that the proposed approach was able to gain some important knowledge about the nature of the program under test for the objective to utilize this knowledge to empower the process of software testing. Therefore, making Assertion-Based software testing more efficient and effective by investing testing resources in those parts of the program that are mostly important to its functionality.

In addition to the “importance” criterion, the proposed approach presented in this paper considers the “confidence” criterion to improve the performance of Assertion-Based software testing. Therefore, in the next step, this approach repeats same process of classifying program's P according to the “confidence” data obtained from the developers as follows. To obtain the “confidence” for this example program, Boyer-Moore, developers were polled to express their confidence in the correctness of this specific program. The result is shown in the first table labeled, “Boyer-Moore,” in Table 3. Using the data obtained in this table, using the *S*-function, we construct the fuzzy set CONFIDENCE as follows. First, we assign the values for the *S*-function parameters: *α*, *β*, and *γ*. As pointed out in [4], Assertion-Based software testing is meant to be applied as complimentary step after traditional testing has been performed to the software, and the confidence in the correctness of the software cannot be too low. Therefore, we set *α* parameter to 20. Similarly, because of the nature software development, nobody can claim that a program is 100% correct and faults-free. Therefore, we set the *γ* parameter to 80. Based on these values of *α* and *γ* parameters, *β* parameter is computed as (*α* + *γ*)/2 = 50. Consequently, the CONFIDENCE fuzzy set is constructed as follows:

 CONFIDENCE = {0/Unit_1, 0.9/Unit_2, 0.5/Unit_3, 1.0/Unit_4}.

The article "Using Fuzzy Logic Techniques for Assertion-Based Software Testing Metrics" was published in 2015. Journal: ScientificWorldJournal.

The values in the CONFIDENCE fuzzy set may be interpreted as follows. The developers have no confidence at all in the correctness of Unit_1. All developers are highly confident that Unit_2 and Unit_4 are fault-free and may not need further tests, while they expressed only 50% confidence in the correctness of Unit_3. Based on the results of this analysis, the proposed approach will concentrate on those programs unit that have low values of in the membership of the CONFIDENCE fuzzy set. For this example, most allotted testing resources will go to Unit_1, followed by Unit_5. Note that without this knowledge, Assertion-Based testing would have been performed equally to all the units in the program without discrimination.

From this example, it is illustrated how applying the proposed technique for Assertion-Based testing metrics may provide a technical and valuable help for the developer while making her decisions about applying Assertion-Based software testing on her software. Additionally, the developer is able to direct their valuable testing resources and efforts towards those parts of the software that are considered to be mostly important and may require additional tastings. As a result of applying the proposed approach, Assertion-Based testing will only be applied to some selected units instead of applying this method to the whole software. The results of this is that the proposed approach will only explore some of the assertions found in the program as compared to exploring all assertions when Assertion-Based testing is applied blindly to the whole software. Therefore, saving valuable search resources, especially when testing programs with large numbers of assertions.

The article "Using Fuzzy Logic Techniques for Assertion-Based Software Testing Metrics" was published in 2015. Journal: ScientificWorldJournal.

## 5. Experimental Study

To evaluate the performance of the proposed technique for Assertion-Based testing metrics, we have performed an experiment. The main objective of this experiment is to show that the proposed technique may be utilized to direct testing resources towards those spots of the programs that need more testing. This experiment is designed as follows. We have asked three programmers to write ten different programs [15] such that each program is composed of several units. Those programs represent an implementation of well-known string searching algorithms [27] reported in the literature.

In the first stage of this experiment, we have seeded some program faults in these programs. After that, we subjected all of the programs to black-box and white-box testing techniques [9]. Specifically, boundary value analysis and equivalence class partitioning and branch coverage testing were performed on those programs. In order to increase our confidence in the correctness of these programs, in the third stage of this experiment, we inserted a number of assertions in each of the programs [4]. At this stage, we performed Assertion-Based testing as reported in [4] on all of the programs with a search time limit of five minutes for each program. Note that Assertion-Based testing that is applied in this stage is as presented in [4] which treats all assertions found in the program equally and will try to violate them one by one sequentially until the allocated search time limit expires. As mentioned previously in Section 2, the objective of Assertion-Based software testing is to generate program input data in order to violate assertions found in the program; if such an input can be generated then this implies that errors exist in the program [4]. The result of this stage is shown in the fourth column of Table 2.

In the fourth stage of this experiment, we have asked the programmers to express their confidence on the correctness of their programs according to the proposed testing metrics technique presented in Section 4. Table 3 shows how the programmers expressed their confidence on the correctness of their programs. Using this knowledge as expressed by the programmers, Assertion-Based testing is performed again on the programs used in this experiment. The result of this stage is shown in the fifth column of Table 2.

The article "Using Fuzzy Logic Techniques for Assertion-Based Software Testing Metrics" was published in 2015. Journal: ScientificWorldJournal.

Table 2 may be interpreted as follows. The first and second columns show the name of the program and the number of units in each program, respectively. The third column shows the total number of assertions in each program. The fourth column reports the number of assertions violated as a result of applying Assertion-Based software testing before considering the testing metrics technique proposed in this paper. The fifth column reports the performance of Assertion-Based software testing as a result of applying the proposed testing metrics technique. For example, in the first row of Table 2, a program named “Boyer-Moore” consists of four units and there were 14 assertions inserted in this program. Applying Assertion-Based testing on this program without considering the proposed approach has resulted in the violations of three assertions as shown in the fourth column of Table 2. After applying the proposed testing metrics technique, two more assertions were violated in this program. This result is reached, by Assertion-Based testing, after considering the recommendations of the proposed testing metrics approach to concentrate on searching Unit_1 and Unit_3 of the program. These recommendations are based on the low confidence points expressed by the developer in Unit_1 and Unit_3 of program “Boyer-Moore” as shown in Table 3. In this specific example, applying the proposed testing metrics technique has resulted in an improvement of 67% in the performance of Assertion-Based software testing. We estimated this improvement percentage as the ability of Assertion-Based testing to violate more assertions in the program. In this experiment, the improvement in the performance of Assertion-Based testing was achieved by giving this approach more time to search for test data to violate assertions.

As indicated by the results of this experiment, applying the proposed testing metrics technique has resulted in an improvement in the performance of Assertion-Based testing as measured by this approach ability to violate more assertions as compared to the case before applying the proposed technique. This encouraging result indicates that using the proposed testing metrics technique has enhanced the performance of Assertion-Based testing by making it utilizes allocated testing resources and to concentrate on violating assertions in certain parts of the program instead of wasting these valuable resources trying to violate all assertions found in the program.

## 6. Conclusions and Future Work

In this paper, we presented a novel software testing metric technique for Assertion-Based software testing that is based on fuzzy logic technology. The main goal of the proposed approach is to enhance the performance of Assertion-Based software testing in the presence of large number of assertions. Furthermore, this approach assists software developers while making their decisions on applying Assertion-Based software testing to their software. In order to evaluate the proposed technique, we have conducted an experimental study in which this technique was applied on a set of programs with assertions. The results of this experiment is very encouraging where applying the proposed approach has enhanced the performance of Assertion-Based testing as shown by the increase on the number of assertions violated in the programs considered in the experiment. In the future, we intend to perform more experiments to evaluate the performance of the proposed technique while applying on commercial size software with large numbers of assertions.

The article "Using Fuzzy Logic Techniques for Assertion-Based Software Testing Metrics" was published in 2015. Journal: ScientificWorldJournal.

## Figures and Tables

**Algorithm 1:** A sample Java method with assertions.

**Table 1:** Data gathered for an example program.

	Unit_1	Unit_2	Unit_3	Unit_4
Developer_A	20%	50%	100%	85%
Developer_B	30%	55%	85%	80%
Developer_C	40%	65%	90%	75%

Average	30%	57%	92%	80%

**Table 2:** Statistics of assertion violations.

Program's name	Number of units	Number of assertions	Assertion violations *before* metrics	Assertion violations *using* proposed metrics technique	Improvements percentage
Boyer-Moore	4	11	3	5	67%
Raita	4	10	1	2	100%
CSA	5	13	3	5	67%
Horespool	3	12	4	6	50%
KR	4	14	3	5	67%
AXAMAC	3	12	3	4	33%
Morris_Patt	4	17	4	5	25%
Quick_Reverse	3	10	2	2	0%
Smith's	3	11	3	5	67%
COLUSSI	5	18	4	6	50%

**Table:** (a) Boyer-Moore

Unit name	Number of assertions	Confidence level
Unit_1	4	20%
Unit_2	3	70%
Unit_3	2	50%
Unit_4	2	80%

**Table:** (b) Raita

Unit name	Number of assertions	Confidence level
Unit_1	2	80%
Unit_2	3	80%
Unit_3	2	70%
Unit_4	3	80%

**Table:** (c) CSA

Unit name	Number of assertions	Confidence level
Unit_1	3	80%
Unit_2	3	80%
Unit_3	3	30%
Unit_4	2	20%
Unit_5	2	80%

**Table:** (d) Horespool

Unit name	Number of assertions	Confidence level
Unit_1	4	30%
Unit_2	4	80%
Unit_3	4	40%

**Table:** (e) KR

Unit name	Number of assertions	Confidence level
Unit_1	5	30%
Unit_2	3	60%
Unit_3	3	80%
Unit_4	3	80%

**Table:** (f) AXAMAC

Unit name	Number of assertions	Confidence level
Unit_1	4	80%
Unit_2	4	50%
Unit_3	4	80%

**Table:** (g) Morris_Patt

Unit name	Number of assertions	Confidence level
Unit_1	5	40%
Unit_2	3	70%
Unit_3	4	80%
Unit_4	5	30%

**Table:** (h) Quick_Reverse

Unit name	Number of assertions	Confidence level
Unit_1	3	80%
Unit_2	3	50%
Unit_3	4	80%

**Table:** (i) Smith's

Unit name	Number of assertions	Confidence level
Unit_1	5	40%
Unit_2	4	50%
Unit_3	2	80%

The article "Using Fuzzy Logic Techniques for Assertion-Based Software Testing Metrics" was published in 2015. Journal: ScientificWorldJournal.

**Table:** (j) COLUSSI

Unit name	Number of assertions	Confidence level
Unit_1	6	50%
Unit_2	5	50%
Unit_3	3	80%
Unit_4	2	80%
Unit_5	2	70%

## References

[1] Korel B. (1990). Automated software test data generation. *IEEE Transactions on Software Engineering*.

[2] Korel B. (1992). Dynamic method for software test data generation. *Journal of Software Testing, Verification, and Reliability*.

[3] Ferguson R., Korel B. (1996). The chaining approach for software test data generation. *ACM Transactions on Software Engineering and Methodology*.

[4] Korel B., Al-Yami A. Assertion-oriented automated test data generation.

[5] Wu X., Sun J. The study on an intelligent general-purpose automated software testing suite.

[6] Karnavel K., Santhoshkumar J. Automated software testing for application maintenance by using bee colony optimization algorithms (BCO).

[7] Srivastava P. R., Baby K. Automated software testing using metahurestic technique based on an Ant Colony Optimization.

[8] Mitra P., Chatterjee S., Ali N. Graphical analysis of MC/DC using automated software testing.

[9] Myers G. (1979). *The Art of Software Testing*.

[10] Zadeh L. A. (1965). Fuzzy sets. *Information and Computation*.

[11] Rafi D. M., Moses K. R. K., Petersen K., Mäntylä M. V. Benefits and limitations of automated software testing: systematic literature review and practitioner survey.

[12] Rosenblum D. S. (1995). Practical approach to programming with assertions. *IEEE Transactions on Software Engineering*.

[13] Alakeel A. M. (2010). An algorithm for efficient assertions-based test data generation. *Journal of Software*.

[14] Shrestha K., Rutherford M. J. An empirical evaluation of assertions as oracles.

[15] Alakeel A., Mhashi M. (2012). Application of intelligent assertion-based testing in string matching algorithms. *The American Journal of Scientific Research*.

[16] Khalid S., Zimmermann J., Corney D., Fidge C. Automatic generation of assertions to detect potential security vulnerabilities in C programs that use union and pointer types.

[17] Alakeel A. Intelligent assertions placement scheme for string search algorithms.

[18] Pezze M., Young M. (2008). *Software Testing and Analysis: Process, Principles and Techniques*.

[19] Nguyen T. B., Delaunay M., Robach C. Testing criteria for data flow software.

[20] Lun L. J., Chi X. Path numbers analysis of relationships on software architecture testing criteria.

[21] Jiang M., Munawar M. A., Reidemeister T., Ward P. A. S. (2011). Efficient fault detection and diagnosis in complex software systems with information-theoretic monitoring. *IEEE Transactions on Dependable and Secure Computing*.

The article "Using Fuzzy Logic Techniques for Assertion-Based Software Testing Metrics" was published in 2015. Journal: ScientificWorldJournal.

[22] Lun L., Chi X. Relationship on path coverage criteria for software architecture testing.

[23] Debbarma M. K., Kar N., Saha A. Static and dynamic software metrics complexity analysis in regression testing.

[24] Rutherford M. J., Carzaniga A., Wolf A. L. (2008). Evaluating test suites and adequacy criteria using simulation-based models of distributed systems. *IEEE Transactions on Software Engineering*.

[25] Singh Y., Kaur A., Malhotra R. (2009). Empirical validation of object-oriented metrics for predicting fault proneness models. *Software Quality Journal*.

[26] Giarratano J. (1989). *Expert Systems: Principles and Programming*.

[27] Stephen G. A. (1994). *String Searching Algorithms*.

[28] Alakeel A. M. Assertion-based software testing metrics approach based on fuzzy logic.

